The article "Integration of Green Innovation Capabilities of Enterprises Based on Ant Colony Optimization Algorithm" was retracted in 2023. Reasons: unreliable results or conclusions; concerns about the data; concerns about the peer review; concerns about the citations.

# Integration of Green Innovation Capabilities of Enterprises Based on Ant Colony Optimization Algorithm

**DOI:** 10.1155/2022/8428641

**Published:** 2022-06-27

**Authors:** Hailin Yang, Fengming Liu, Lihong Zhang

**Affiliations:** ^1^School of Business, Shandong Normal University, Jinan 250358, Shandong, China; ^2^School of Political Science and Law, Qilu University of Technology (Shandong Academy of Sciences), Jinan 250353, Shandong, China

## Abstract

This article studies the integration and optimization of green innovation capabilities of enterprises. The integration model of enterprise green innovation capability provides the theoretical basis for cultivating enterprise green innovation capability. However, from the perspective of optimization, in the life cycle of the enterprise, how the enterprise should reasonably allocate resources and carry out strategic guidance to achieve the optimal green innovation capability of the enterprise is a question worth thinking about. This stage of research starts from different cycle stages of enterprise development, explores the adaptability and evolution of the integration model, and studies the optimization methods of strategies to achieve the goal of matching. This article adopts the ant colony optimization algorithm to support the research on the integration of green innovation capabilities of enterprises. The article describes the principle of the ant colony optimization algorithm in detail by using the combination of text description and formula. In addition, it analyzes the effect of the research through experiments. The results show that the corresponding CITC coefficients of each item of the Green Innovation Scale are between 0.518 and 0.850, which are all greater than the ideal value of 0.4.

## 1. Introduction

The innovation-driven strategy is the top priority of China's strategy, and as the driver of the national economy, enterprises shoulder huge responsibilities and missions, so the development of enterprises is very important. In this case, as a value-added system, the creativity of the enterprise depends on the integration of different subjects, elements and resources in the enterprise, so that each value link can be optimized and the overall performance of lasting innovation ability. However, looking at the relevant research on the green innovation capabilities of Chinese enterprises, it mainly continues the research ideas of other countries, ignoring the endogenous driving force of the integration of enterprises' green innovation capabilities, and lacks research on enterprises' green innovation capabilities from the perspective of the complex adaptability of system evolution. In particular, there are very few studies based on the concept of innovation ecology.

The article "Integration of Green Innovation Capabilities of Enterprises Based on Ant Colony Optimization Algorithm" was retracted in 2023. Reasons: unreliable results or conclusions; concerns about the data; concerns about the peer review; concerns about the citations.

This paper will use the theories of ecology, system theory, evolutionary view, integration thinking and other theories to conduct in-depth research on the green innovation capability of enterprises. This will expand the existing research ideas and add new branches to the innovation research system, which will also deepen knowledge management theory and enterprise innovation theory. At the same time, the research on enterprise green innovation system and its evolution in this article is exactly the real problem faced by enterprise construction now. These research results will provide meaningful suggestions for the practice of enterprise innovation projects and the cultivation of enterprises' sustainable innovation ability.

(2) This article will use the theories of ecology, system theory, evolutionary view, integration thinking, and other theories to conduct in-depth research on the green innovation capability of enterprises. This will expand the existing research ideas and add new branches to the innovation research system, deepening knowledge management theory and enterprise innovation theory. At the same time, the research on enterprise green innovation system and its evolution in this article is exactly the real problem faced by enterprise construction now. These research results will provide meaningful suggestions for the practice of enterprise innovation projects and the cultivation of enterprises' sustainable innovation ability.

## 2. Related Work

Many scholars have provided a lot of references for the research on ant colony optimization algorithm, capability integration, and green innovation capability of enterprises.

Zhou and Cao discussed the evolution of green innovation in Chinese coal companies and the various driving mechanisms that are affected by government regulations, corporate resource capabilities, and supply chain integration [1].

Rossiter and Smith analyzed sustainable housing developments in the UK city of Nottingham in the form of not only sustainable housing projects but also experiments in developing sustainable communities. In terms of green or ecological innovation, it combines innovations in housing design aimed at curbing energy demand; innovations in energy supply technologies centered on new community energy systems; innovations in the governance models employed [2].

Qiu et al. focused on how green product innovation affects the green power capability and competitive advantage of Chinese manufacturing. Qiu et al. also found that the resource integration ability, resource reconstruction ability, and environmental insight ability of green power capability play a mediating role between green product innovation and competitive advantage [3].

The article "Integration of Green Innovation Capabilities of Enterprises Based on Ant Colony Optimization Algorithm" was retracted in 2023. Reasons: unreliable results or conclusions; concerns about the data; concerns about the peer review; concerns about the citations.

Ardyan et al. examined green innovation capabilities as a driver of sustainable competitive advantage and SME marketing performance. The research results show that green innovation ability can significantly improve sustainable competitive advantage, and sustainable competitive advantage can significantly improve the marketing performance of SMEs [4].

Salunke et al. examined the role of the antecedents of knowledge integration capabilities (KIC) in service innovation-led competitive advantage in project-oriented B2B service firms. They modeled and empirically tested the link between KIC and service innovation and then tested sustainable competitive advantage (SCA) [5].

Bo et al. proposed a theoretical model to study the antecedents and consequences of elastic and plastic innovation capabilities. The findings suggest that a firm's past performance is positively correlated with its ability to innovate resiliency. Elastic innovation ability and organizational willingness are positively related to plastic innovation ability. The innovative capabilities of elasticity and plastics significantly lead to superior performance [6].

Zheng et al. proposed an innovative parameter adaptation strategy for Ant Colony Optimization (ACO) algorithm. The strategy is based on controlling the convergence trajectory in the decision space to follow any prespecified path, aiming to find the best possible solution given and a limited computational budget [7].

The data of these studies are not comprehensive, and the results of the studies are still open to question, so they cannot be recognized by the public and thus cannot be popularized and applied.

## 3. Integration of Green Innovation Capabilities of Enterprises

Foraging is a collective behavior of ants. On the way of foraging, each ant chooses where to move through the pheromone released by other ants and leaves a corresponding number of pheromones on the path it travels. These pheromones can be sensed by other ants and slowly evaporate over time. The number of pheromones represents the distance to the food source: the larger the number, the closer to the food source; the smaller the number, the farther to the food source. Under normal circumstances, ants will go to the road with more pheromone with greater probability and then release a certain amount of pheromone on this road to increase the concentration of pheromone on this path. This provides positive feedback to other ants, and finally, the ant colony will find a path closest to the food source [8, 9].

The ACO algorithm can study many combinatorial optimization problems. We can take a path traversed by ants as a correct solution to the optimization problem, then the feasible path obtained is the solution space of the problem to be optimized. Ants secrete more pheromones on short-distance roads, so as other ants explore the road, the concentration of pheromone secreted on closer roads will be higher, and then more ants will appear on this road. As a result, under the influence of this positive feedback mechanism, ants will concentrate on an optimal path to reach the food source so that the combinatorial optimization problem is solved [10, 11].

The article "Integration of Green Innovation Capabilities of Enterprises Based on Ant Colony Optimization Algorithm" was retracted in 2023. Reasons: unreliable results or conclusions; concerns about the data; concerns about the peer review; concerns about the citations.

Based on the process of the ant colony algorithm solving optimization problems, compared with other intelligent optimization algorithms, it is not difficult to see some advantages of the ant colony algorithm:

1. Information positive feedback mechanism [12, 13]: this mechanism can make the ant's search process converge continuously and obtain the best solution after repeated cycles [14].
2. The release and volatilization of pheromones [15]: each ant can change the surrounding environment by releasing pheromone and indirectly convey information to other companions, and the volatilization of pheromones can speed up the determination of the optimal path [16, 17].
3. Distributed computing [18]: multiple individuals of the ant colony search for paths at the same time. This distributed method can improve the calculation speed of the algorithm and increase the operating efficiency [19, 20].
4. Heuristic exploration [21]: when each ant finds a path, heuristic exploration is carried out according to the heuristic factor, which can prevent the result from falling into the local optimum, and is beneficial to obtaining the global optimum solution of the optimization problem [22, 23].

In order to improve the application performance of the ACO algorithm in the network, some researchers improve the pheromone mechanism of the basic ACO algorithm in the SDN environment and divide the pheromone in the algorithm into foraging pheromone (FP) and tracking pheromone (TP). When the ant is looking for the next node, it will judge which pheromone to rely on according to the type of node it is located. When the ant reaches an overloaded node, the ant will follow the pheromone and update the TP trace of the path. When reaching a low-load node of the same type, in order to transfer the data of the overloaded node to the low-load node, they will update the data structure and then freely select an adjacent node to repeat the above process, thereby improving the performance of the network. This improvement can cope well with the situation of node state flipping and improve the stability of the network.

The article "Integration of Green Innovation Capabilities of Enterprises Based on Ant Colony Optimization Algorithm" was retracted in 2023. Reasons: unreliable results or conclusions; concerns about the data; concerns about the peer review; concerns about the citations.

Multi-ant colony optimization algorithm (MACO) uses multiple ant colonies to deal with combinatorial optimization problems and is an improvement direction of the ant colony optimization algorithm. Pheromone is the medium of cooperation among multiple ant colonies, and each ant colony has its own pheromone. The basic ACO algorithm only uses a positive pheromone feedback mechanism, while MACO considers both positive and negative pheromone so that ants can share information with each other so that the ants have more space for exploration. The algorithm is applied to the task scheduling load balancing problem, and its performance is obviously stronger than the algorithm of a single ant colony system. Moreover, MACO takes the average number of pheromones as the standard and has good performance in dealing with large-scale cases.

From the beginning to deal with the traveling salesman problem (TSP) to the later wireless sensor network, cloud computing task allocation, and other problems, the ACO algorithm has shown a good processing effect. Compared with other bionic intelligent optimization algorithms, the time to use it to get the best results is shorter.

The concept of ecological niche refers to the sum of the status and status of species in the ecosystem. With the introduction of the ecological method into the research of technological innovation clusters, the concept of enterprise niche is proposed. It refers to the position and status of the enterprise in the cluster environment and the relationship with other enterprises, which determines the sum of the enterprise's use of the resources in the cluster and the adaptation to the cluster environment. The enterprise niche contains many different resource dimensions, and the enterprise's utilization capability and selection range in each resource dimension constitute a set of complex relationships, which is the structure of the enterprise niche. In fact, as an innovation ecosystem, the core of an enterprise is the collaborative innovation of knowledge. The concept of knowledge niche can only be understood when we examine the generation and evolution of this innovative ability from the perspective of knowledge management and niche integration. The key to understanding the knowledge niche is understanding the division of knowledge categories in the innovation ecosystem.

Because the innovation ecological chain network of enterprises is a complex system based on the division of enterprise knowledge, with the interaction of different knowledge subjects and knowledge innovation as the core, it is very necessary to study the innovation ability of different knowledge subjects and the whole system from the perspective of “knowledge niche.” Based on the division of knowledge categories in innovation and the corresponding concept of enterprise niche, this article argues that knowledge niche is the sum of auxiliary knowledge and complementary knowledge occupied by enterprises. The content of complementary knowledge that an enterprise occupies in an innovation chain means the degree of specialization of its core knowledge in this link in the chain, which represents the depth of the enterprise's knowledge niche. The auxiliary knowledge has the characteristics of generality and high redundancy. How much it is occupied by enterprises determines the boundaries of knowledge that enterprises can use and represents the breadth of enterprise knowledge niches. Therefore, the depth and breadth of knowledge niches form the unique knowledge space of enterprises. Knowledge niche overlap reflects the intersection of knowledge niches among firms, which obviously depends on the breadth of auxiliary knowledge. The knowledge niche overlap density reflects the overlap of all enterprises in a certain link in the knowledge niche, and it depends on the breadth of the auxiliary knowledge of each enterprise and the number of competing enterprises in the same link.  Figure 1 illustrates the knowledge niches of specialized and generalized firms.

The article "Integration of Green Innovation Capabilities of Enterprises Based on Ant Colony Optimization Algorithm" was retracted in 2023. Reasons: unreliable results or conclusions; concerns about the data; concerns about the peer review; concerns about the citations.

The enterprise knowledge niche is always in dynamic change, and the overlap and separation of knowledge niche among enterprises are also in dynamic evolution. As more and more auxiliary knowledge content is required for innovation among enterprises, the overlapping parts of knowledge niches among enterprises will become more and more. Externally, it may manifest as similar product structure, technological innovation path, institutional structure, demand space, etc. When the overlap exceeds a certain level, it may cause fierce competition among enterprises in the same link in the industrial chain, and there are few opportunities for cooperation. In the vertical structure of the industrial chain, enterprises in certain links are annexed by upstream and downstream links, and the living space is greatly squeezed. On the contrary, when an enterprise deepens its ability to utilize a certain knowledge resource in order to avoid competition, the enterprise's knowledge niche will be separated from other enterprises, and it will protect its own knowledge niche and even open up a potential knowledge niche for exclusive use. But at this time, the innovation of enterprises basically relies on their own core knowledge and seldom considers complementary cooperation. Therefore, if the enterprises in the cluster want to achieve the maximum innovation efficiency in a short period of time by means of integrated innovation, the enterprises need to maintain a suitable degree of overlapping of knowledge niches, thereby increasing the opportunities for enterprises to carry out collaborative innovation, reducing the innovation cost of enterprises, and enabling enterprises to find the most suitable partners. Adopting the strategy of “mutual benefit and symbiosis,” expand the knowledge niche through integration, enhance “survival ability,” and achieve “win-win.” Of course, the appropriate degree of niche overlap is not fixed but changes from time to time.  Figure 2 illustrates that under the appropriate degree of knowledge niche overlap, the common knowledge niche is expanded through synergistic integration among firms.

The article "Integration of Green Innovation Capabilities of Enterprises Based on Ant Colony Optimization Algorithm" was retracted in 2023. Reasons: unreliable results or conclusions; concerns about the data; concerns about the peer review; concerns about the citations.

In the enterprise innovation system, from the perspective of the innovation chain, the innovation of an enterprise not only comes from the pull of innovation by upstream and downstream enterprises in the vertical industrial chain, the promotion of cooperation between enterprises, and the imitation competition of horizontal similar enterprises and the cooperation of complementary enterprises. It also includes collaborative innovation on the knowledge chain formed by enterprises, universities, R&D institutions, and other knowledge institutions. Combined with the interpretation of the connotation of knowledge niche integration, the essence of enterprise green innovation capability integration is the integration of knowledge niche between enterprises through collaborative innovation. However, it should be noted that different ways of integrating knowledge niches result in different innovation capabilities. Each enterprise occupies a different knowledge niche as a different knowledge subject. In the process of collaborative innovation, the types of innovations generated by the interaction of knowledge niches are not the same. According to the dual view of innovation classification, the green innovation capability of enterprises can be divided into incremental innovation and breakthrough innovation. Incremental innovation is localized and improved innovation with the accumulation of knowledge and technology. Breakthrough innovation is a fundamental change to the product due to the fusion of advantageous knowledge between different organizations. In the process of collaborative innovation, when the innovation cooperation between enterprises is aimed at improving innovation, the cognitive distance of knowledge between enterprises is small, and knowledge is easy to transfer and understand. At this time, the knowledge exchanged between enterprises is mostly auxiliary knowledge. When the innovation cooperation between enterprises is aimed at breakthrough innovation, the knowledge among enterprises is mainly complementary knowledge based on certain common knowledge. Although the cognitive distance between enterprises is large at this time, knowledge is not easy to understand and integrate, but this can stimulate the learning potential of each organization. Through the collision, integration, and reconstruction of knowledge, breakthrough innovation can often be produced at this time.

The article "Integration of Green Innovation Capabilities of Enterprises Based on Ant Colony Optimization Algorithm" was retracted in 2023. Reasons: unreliable results or conclusions; concerns about the data; concerns about the peer review; concerns about the citations.

Enterprise green innovation system and natural ecosystem have similar characteristics. Enterprise members form technological innovation chain, technological innovation network, and technological innovation community based on the division of labor and cooperation, which are similar to the food chain, food web, and community in the ecosystem. The basic structure of the innovation system is hierarchical and modular (as shown in Figure 3). As can be seen from Figure 3, the hierarchy is manifested in that with the extension of the industrial chain, enterprises are in different links, forming a vertical division of labor. Moreover, there is not only one enterprise but multiple enterprises in each link, and these enterprises will continue to form derivative chains in the same link. It may be a complementary relationship, a matching relationship, etc. Modularity is manifested in that when a core enterprise drives the cooperation of supporting enterprises, it is necessary to form consistent technical standards and technical interfaces. At this time, each enterprise as a technical module is well coupled based on the same standard.

The specific definitions of the influencing factors of enterprise innovation capability have three types are innovation input, innovation environment, and innovation output, as follows:

1. Innovation investment: innovation input is the source of power for innovation subjects to carry out innovation activities. If there is a lack of innovation investment, the development of the enterprise will be insufficient due to a lack of motivation, the green innovation capability of the enterprise will be difficult to improve, and the enterprise innovation may face failure. The strength of an enterprise's innovation investment capability is usually measured by indicators such as input personnel, funding expenditure, and scientific research resources. The input personnel reflects the allocation of innovative talents in the main innovation activities in the enterprise and is an important indicator to measure whether the innovation subject has innovation potential. Expenditures reflect the financial support required by innovative entities in the enterprise for R&D and innovation, and it provides sufficient power for innovative entities to conduct R&D and innovation. Scientific research resources reflect the research and development capabilities of innovative entities within an enterprise and indirectly indicate the development level of enterprise innovation.
2. Innovation environment: the innovation environment generally refers to the external environment in which the innovation subject conducts innovation activities, including the development level of the Internet, the popularization of information, and the support of the government, finance, intermediary services, and other institutions. The success of the innovation activities of the innovation subject is closely related to the external environment in which it is located. A good external environment is a key factor in improving the innovation ability of the innovation subject. The innovation environment is mainly reflected by the degree of informatization, government support, financial environment, and Internet development. The degree of informatization reflects the interaction and exchange of innovation subjects among enterprises, and government support reflects the degree of government agencies' support for enterprise innovation activities. The financial environment reflects the degree of support of financial institutions to the innovation activities of enterprises, and the level of Internet development reflects the openness of the environment in which enterprises are located, which can provide various required information for enterprise innovation.
3. Innovation output. The innovation output mainly refers to the ability of the innovation subject to transform the innovation input into various scientific research achievements in the innovation process, which most directly shows the actual effect of the innovation subject's innovation activities. If the innovation subject has many scientific research achievements and high transformation efficiency, it can not only arouse the interest of other innovation subjects in scientific and technological innovation but also encourage other innovation elements to gather in this enterprise. This will provide sufficient impetus for the innovation and development of the enterprise and form a favorable situation of interaction and cooperation among innovation entities within the enterprise and a virtuous circle of resource elements. Innovation output is mainly measured from two aspects: direct innovation results and technology transfer and cooperation. The direct result of innovation is the direct manifestation of the innovation output of the enterprise, and technology transfer and cooperation reflect the collaboration and exchange of the innovation output of the innovation main body of the enterprise.
4. Complete openness is the precondition for the evolution of the enterprise innovation system. If the enterprise innovation system wants to develop by leaps and bounds, it is essential to continuously obtain energy from the external environment, and this also requires the enterprise innovation system to remain fully open. Only under the premise of full opening can the enterprise innovation system be able to fully understand the market demand and competition conditions and can promote the economic growth of the enterprise lastingly. Otherwise, standing still will only lead to “innovation” unable to create due value and eventually be gradually eliminated in the market competition.
5. Far from equilibrium is the power source of the evolution of enterprise innovation system. An enterprise innovation system far from equilibrium means that there are significant differences in the specialization of labor, resource allocation, and fixed investment within the system. These differences can fully mobilize the innovation enthusiasm of the scientific and technological personnel in the system and provide a guarantee for the realization of innovation and the productization of innovation. If the enterprise innovation system is in a balanced state as a whole, it will not be able to gain insight into the rapidly changing market demands in a timely manner, and the entire system will be gradually eliminated in the fierce market competition. Therefore, in the process of system development, each innovation subject and subsystem must constantly change and form unique advantages or differences.
6. Small fluctuations are the direct cause of the evolution of enterprise innovation system. There are many small fluctuation factors in the enterprise innovation system. Changes in policies and regulations, technological innovation and development, financial market fluctuations, market demand changes, and consumer demand changes will all have an impact on the ups and downs of the corporate innovation system. When many small fluctuations gradually accumulate to form a huge scale effect, that is, small fluctuations form giant fluctuations, the entire enterprise innovation system will undergo huge changes. That is to say that these small fluctuations are the driving factors that break the original equilibrium state of the enterprise innovation system.
7. Nonlinear action is the fundamental guarantee for the evolution of enterprise innovation system. The role of each subject and each subsystem of the enterprise innovation system is nonlinear. The various subjects and subsystems within the system maintain contact and restrict each other through nonlinear effects such as competition, cooperation, and coordination and integrate resources through communication and cooperation. These so-called linkages and constraints refer to the cyclical influence between two or more parties, thereby producing interactive and synergistic effects between various subjects and subsystems so as to promote the transformation of the enterprise innovation system from a low-level order to a high-level order.
8. The self-organization evolution of enterprise innovation system is a process from disorder to order, from backward to advanced, from nothing to existence, from existence to excellence. In this process, the system can spontaneously exchange and flow material, information, and energy without an external push. And under the nonlinear action, many tiny fluctuations in the system gradually enlarge into giant fluctuations, resulting in new qualitative changes, breaking the stable state of the system, and the system begins to transform from a disordered state to an ordered state. Such cyclical and repeated transformations make the system eventually tend to a stable state, which constitutes the self-organized evolution process of the entire system. It is generally believed that each round of self-organization evolution of an enterprise innovation system needs to go through three stages, namely, the stable and disordered stage, the unstable stage, and the new stable and orderly stage.
9. Stable disorder stage: at this stage, although the system is in a stable state, there are still the exchange and flow of matter, information, and energy in it, but there is a lack of inducing factors that cause the system changes. Once the inducement factors appear, the system will face the end of the disordered and stable stage, that is, the beginning of the system's small fluctuations, and the entire enterprise innovation system will undergo great changes. This also means that the appearance of inducing factors breaks the original disordered and stable state of the system, and the system begins to generate fluctuation factors in the process of exchange of matter, information, and energy. These fluctuation factors can be internal factors (changes in policies and regulations, innovations in business management methods, etc.) or external factors (development of science and technology, changes in market demand, etc.).
10. Instability stage: strictly speaking, this stage can be subdivided into the initial instability stage and the complete instability stage. In the initial instability stage, many small fluctuation factors generated in the system begin to play a role, and the main elements and object elements of innovation gradually realize the influence of fluctuations. And the entire system begins to undergo many small changes. In the complete instability stage, once the inducing factors appear, the influence range of the microfluctuation gradually spreads under the complex nonlinear action and finally becomes a giant fluctuation. The influence of giant fluctuations gradually develops to the maximum and affects the entire enterprise innovation system. The enterprise innovation system will face fundamental changes and development, and the system will undergo drastic changes and move toward an orderly direction.
11. New stable and orderly stage: after going through the complete instability stage, the impact of huge fluctuations on the system will stabilize after a period of time, and the enterprise innovation system will stabilize again. At this time, the corporate innovation system will undergo structural changes and become more orderly and stable. After the system undergoes the transformation process from low-level order to high-level order, the new system formed still meets the conditions for self-organizing evolution. Under the action of these conditions, the system will start the self-organizing path evolution process again so as to develop to a higher-order structure.

The article "Integration of Green Innovation Capabilities of Enterprises Based on Ant Colony Optimization Algorithm" was retracted in 2023. Reasons: unreliable results or conclusions; concerns about the data; concerns about the peer review; concerns about the citations.

The integration of knowledge niches generates new knowledge and forms innovation, and the synergy between vertical knowledge ecological chains is closely is related to this innovation. Enterprises are in different links in the vertical knowledge ecological chain, and the knowledge ecological niches they occupy are also different. Generally speaking, in this vertical relationship, the integrated innovation among enterprises in different links is based on the modular structure of the industrial chain. The two types of enterprises in different technical knowledge links occupy significantly different knowledge positions and thus produce different types of innovations (Figure 4).

In the same link of the knowledge ecological chain, due to the continuous division of labor and extension of the knowledge ecological chain, more branch chains have been derived from enterprises in the same link. These chains represent cooperative or multilevel matching relationships. Enterprises in the same link adopt the mode of collaborative innovation to enhance their core competitiveness for greater benefits, thereby optimizing the innovation capability of this link (Figure 5).

The sample descriptive statistics and independent samples test are shown in Tables 1 and 2, respectively.

Table 1 shows that there is a strong positive correlation between the knowledge complementarity of enterprises and other enterprises and the two different types of innovation they exert.

The article "Integration of Green Innovation Capabilities of Enterprises Based on Ant Colony Optimization Algorithm" was retracted in 2023. Reasons: unreliable results or conclusions; concerns about the data; concerns about the peer review; concerns about the citations.

Table 2 shows that companies with general technology modules are more likely to show incremental innovation in the process of collaborative innovation in the industrial chain; proprietary technology modules are more likely to be breakthrough innovations than general technology modules.

After calculating the estimated value of the model for the first time, it was shown that the model could not fit the real data, and the model was rejected. Based on combining model correction indicators and theories by deleting insignificant paths in the model, adding new path relationships, and grasping the principle of changing only one place for each modification so as to avoid model distortion after a large-scale modification, after several rounds of modification, a modified model that matches the actual data well is obtained. The quality parameters of the measured model in the revised model are shown in Tables 3–5.

Tables 3–5 show that enterprise knowledge fusion ability has a significant positive impact on incremental innovation. The knowledge integration capability of an enterprise means whether an enterprise can integrate the absorbed knowledge into its own knowledge system and transform it into knowledge useful for innovation. This is the core capability of an enterprise's knowledge niche integration capability. But at the same time, it should be noted that in the surveyed area, this ability often has a significant positive effect on the incremental innovation ability in the innovation ability but has no significant effect on the breakthrough innovation ability.

## 4. Ant Colony Optimization Algorithm

The ACO algorithm is a bionic algorithm obtained by simulating the inspiration of ant groups in the biological world to find food. Ants transmit information to their remaining companions by virtue of the hormones secreted on the road they crawl, so the models of basic ACO algorithms are built around pheromones.

The probability of ant *ϖ* at position *μ* choosing position *ν* is as follows:

(1) $$\begin{array}{c} p_{\mu \nu }^{\varpi }=\frac{\tau_{\mu \nu }^{\alpha }\eta_{\mu \nu }^{\beta }}{\sum_{\nu \in A}\tau_{\mu \nu }^{\alpha }\eta_{\mu \nu }^{\beta }}. \end{array}$$

Among them, *ϖ* is the number of the ant colony individual, *μ* is the current position of the ant colony individual, and *ν* is the position that the ant colony individual can choose. *A* is the set of the ant's next optional position above and below position *μ*, *τ*_*μν*_ is the pheromone concentration between positions *μ* and *ν*, *η*_*μν*_ is the visibility of positions *μ* and *ν*, and *α* and *β* are the weights of pheromone concentration and visibility, respectively, which represent the influence of the two on the ant's choice of location.

The article "Integration of Green Innovation Capabilities of Enterprises Based on Ant Colony Optimization Algorithm" was retracted in 2023. Reasons: unreliable results or conclusions; concerns about the data; concerns about the peer review; concerns about the citations.

The variation of pheromone concentration between positions *μ* and *ν* mainly includes natural evaporation and ant release:

(2) $$\begin{array}{c} \tau_{\mu \nu }\left(\xi +1\right)=\rho *\tau_{\mu \nu }\left(\xi \right)+\sum_{\varpi =1}^{\omega }\Delta \tau_{\mu \nu }^{\varpi }. \end{array}$$

Among them, *ρ* is the pheromone evaporation coefficient of the pathway.

Three calculation models of the amount of pheromone secreted by ant colony individuals on the road are the ant cycle system model, ant quantity system model, and ant density system model.

(3) $$\begin{array}{c} \Delta \tau_{\mu \nu }^{\varpi }=\frac{Q}{L_{\varpi }},\\ \Delta \tau_{\mu \nu }^{\varpi }=\frac{Q}{d_{\mu \nu }},\\ \Delta \tau_{\mu \nu }^{\varpi }=Q. \end{array}$$

Among them, *Q* is the total amount of pheromone released by the individual ant colony, and *L*_*ϖ*_ in the ant cycle system model is the size of the distance ants crawl, and the ants determine the amount of pheromone released according to the length of the global optimal road. In the ant quantity system model, *d*_*μν*_ is the distance between positions *μ* and *ν*, and the ants determine the amount of pheromone released according to the local path length. The ant density system model does not consider the length of the road found by the ants and sets the amount of secreted pheromone as *Q*. In order to ensure the convergence and stability of the algorithm, the ant cycle system model is generally used to calculate the amount of pheromone secreted by ants on the road. The smaller the distance, the more pheromone left by the ants.

The transition rule used by the ants in the ACO algorithm is the roulette method. As shown in Figure 6, the probability that the ants at the current node 1 select nodes 2 and 3 is P(1, 2) and P(1, 3), respectively.

Update the velocity and position of the *μ*-th particle in the *ν*-th dimension in each generation:

(4) $$\begin{array}{c} w_{\mu \nu }\left(\varpi +1\right)=x\left(\varpi \right)w_{\mu \nu }\left(\varpi \right)+d_{1}s_{1}\left(q_{\mu \nu }\left(\varpi \right)-y_{\mu \nu }\left(\varpi \right)\right)+d_{2}s_{2}\left(h_{\mu \nu }\left(\varpi \right)-y_{\mu \nu }\left(\varpi \right)\right),\\ y_{\mu \nu }\left(\varpi +1\right)=y_{\mu \nu }\left(\varpi \right)+w_{\mu \nu }\left(\varpi +1\right),\\ x\left(\varpi \right)=x_{\max}-\frac{x_{\max}-x_{\min}}{\varepsilon_{\max}}\varpi . \end{array}$$

Among them, *d*_1_ and *d*_2_ are learning factors, *s*_1_ and *s*_2_ are [0, 1], *x*(*ϖ*) is the *ϖ*-th generation particle, and *ε*_max_ is the maximum iteration algebra.

The individual best position of particle *μ* is as follows:

(5) $$\begin{array}{c} Q_{\mu }\left(t\right)=\left\{\begin{array}{c} Y_{\mu }\left(t\right)\text{if}f\left[Y_{\mu }\left(t\right)\right]<f\left[Q_{\mu }\left(t-1\right)\right],,\\ Q_{\mu }\left(t-1\right)\text{if}f\left[Y_{\mu }\left(t\right)\right]\geq f\left[Q_{\mu }\left(t-1\right)\right], \end{array}\right.\\ Q_{\mu \nu }\left(t\right)=\phi_{\nu }\left(t\right).Q_{\mu \nu }\left(t\right)+\left[1-\phi_{\nu }\left(t\right)\right].H_{\nu }\left(t\right)\phi_{\nu }\left(t\right)\in U\left(0,1\right). \end{array}$$

Suppose there are *ω* ants searching in the whole world, and the *ω* paths traveled by *ω* ants constitute a genetic population *B*:

(6) $$\begin{array}{c} B=\left[\begin{array}{c} b_{1.1},b_{1.2},\ldots ,b_{1.\nu },\ldots ,b_{1.\xi },b_{2.1},b_{2.2},\ldots ,b_{2.\nu },\ldots ,b_{2.\xi },\ldots \ldots ,\\ b_{\mu .1},b_{\mu .2},\ldots ,b_{\mu .\nu },\ldots ,b_{\mu .\xi },\ldots \ldots ,b_{\omega .1},b_{\omega .2},\ldots ,b_{\omega .\nu },\ldots ,b_{\omega .\xi } \end{array}\right]. \end{array}$$

Let the fitness function be

(7) $$\begin{array}{c} L_{t}=\sum_{\mu =1}^{\xi }d_{l},\;T=1,2,\ldots ,\omega . \end{array}$$

Let the two optimal parents with the best fitness be

(8) $$\begin{array}{c} B=\left[b_{1.1},b_{1.2},\ldots ,b_{1.\nu },\ldots ,b_{1.\xi }\right],\\ B=\left[b_{2.1},b_{2.2},\ldots ,b_{2.\nu },\ldots ,b_{2.\xi }\right]. \end{array}$$

(1) Randomly select an intersection area on the parent string; for example, the two parent strings are
  (9) $$\begin{array}{c} \chi_{1}=12\left|3456\right|789\\ \chi_{2}=98\left|7654\right|321. \end{array}$$
(2) Adding the intersection area of *χ*_1_ to the front of *χ*_2_ and the mating area of *χ*_1_ to the front of *χ*_2_,
  (10) $$\begin{array}{c} \chi_{1}^{\prime }=7456|123456789\\ \chi_{2}^{\prime }=3456|987654321. \end{array}$$
(3) Deleting the same numbers in *χ*_1_′, *χ*_2_′ as the intersection area in turn to get the final two substrings,

(11) $$\begin{array}{c} \delta_{1}=745612389\\ \delta_{2}=345698721. \end{array}$$

After *t* iterations, the increment of the pheromone allocated to each edge on the path traversed by ant *ϖ* is *ϖ*_*μν*_*V*; among them, *ϖ*_*μν*_ is the allocation coefficient, and the increment of the pheromone allocated on the path is *V*=*ξ*/*L*^*ϖ*^(*t*). The specific calculation process is as follows:

(12) $$\begin{array}{c} l_{\mu \nu }=\frac{1}{d_{\mu \nu }},\\ L=\sum_{\left(\omega ,\xi \right)\in B\left(\varpi \right)}\left(\frac{1}{d_{\omega \xi }}\right),\\ \varpi_{\mu \nu }=\frac{l_{\mu \nu }}{L}. \end{array}$$

According to the measurement scale, taking technology-based SMEs as the survey object, a total of 342 pieces of valid data were obtained through questionnaires for empirical analysis. The industry distribution of sample companies is shown in Figure 7.

The article "Integration of Green Innovation Capabilities of Enterprises Based on Ant Colony Optimization Algorithm" was retracted in 2023. Reasons: unreliable results or conclusions; concerns about the data; concerns about the peer review; concerns about the citations.

Figure 7 shows that among the 342 valid questionnaires, there are 112 and 87 new materials and optomechatronics companies, accounting for 32.7% and 25.4% of the total sample size and more than half of the sample size.

The regional distribution of sample companies is shown in Figure 8.

As can be seen from Figure 8, the companies with valid survey data are mainly concentrated in Guangdong, Jiangsu, Zhejiang, Beijing, Shanghai, Shandong, and other places, while the number of surveyed companies in other regions is scattered or even sporadically distributed. This distribution also reflects the current situation of the regional distribution of China's technology-based SMEs; that is, the regional distribution is extremely unbalanced. Guangdong, Jiangsu, Zhejiang, Beijing, Shanghai, Shandong, and other regions with relatively developed economies have more technological SMEs than other regions, while the number of technological SMEs in areas to be developed is also less.

The reliability analysis results of the green innovation influencing factor scale are shown in Figure 9.

Figure 9 shows that the Cronbach's Alpha values of the four variables of government-level influencing factors, enterprise-level influencing factors, market-level influencing factors, and social-level influencing factors are 0.829, 0.864, 0.867, and 0.845, respectively, all greater than 0.8. Moreover, the corresponding CITC coefficients of each item included in the scale are close to or greater than 0.4, and the above indicators indicate that the reliability of the green innovation influencing factor scale is good.

The reliability analysis results of the green dynamic ability scale are shown in Figure 10(a). The reliability analysis results of the green innovation scale are shown in Figure 10(b).

Figure 10(a) shows that the CITC coefficients of all items on the green dynamic ability scale are above 0.598, which are all greater than the ideal CITC coefficient of 0.4. At the same time, the Cronbach's Alpha value of the green innovation capability scale is 0.909, which is also greater than 0.8. In conclusion, the green dynamic capability scale has good reliability. Figure 10(b) shows that the corresponding CITC coefficients for each item of the green innovation scale are between 0.518 and 0.850, which are all greater than the ideal value of 0.4. And the Cronbach's Alpha value of the green innovation scale is 0.844, which is greater than 0.8, so the reliability of the green innovation scale is good.

## 5. Discussion

Enterprises are not only a powerful driving force for local and national economic development but also the birthplace of innovation. It is dominating the world economy today, but Chinese enterprises are exposed to the phenomenon of unsustainable innovation and insufficient dynamic adaptability. They are facing the situation of being locked in technology and need to stand out in the competition with other countries and break through the bottleneck. Based on the concept of innovation ecology, this article conducts in-depth research on how to improve the green innovation capability of enterprises, obtains some meaningful findings, and gives some policy suggestions on the development of enterprises.

The article "Integration of Green Innovation Capabilities of Enterprises Based on Ant Colony Optimization Algorithm" was retracted in 2023. Reasons: unreliable results or conclusions; concerns about the data; concerns about the peer review; concerns about the citations.

First, on the basis of defining the connotations of related concepts such as innovation ecosystem, innovation capability, and knowledge niche, this article uses the mathematical model of game theory to deduce the evolution process of enterprise knowledge niche overlap within an enterprise. This paper expounds the integration mechanism of two different knowledge niches in different links and the same link in the enterprise green innovation system. Secondly, this article comprehensively and systematically analyzes the important factors affecting the innovation capability of enterprises from the dimension of enterprise knowledge niche integration capability and the dimension of green innovation system attributes. Using the method of structural equation modeling, this article constructs a generation model of enterprise innovation ability with good explanatory power through the links of hypothesis, test, and modification and deeply analyzes the generation mechanism of innovation ability in enterprises. Finally, on the basis of the model, combined with the point of view of the enterprise life cycle, from the perspective of dynamics and evolution, the focus and optimization suggestions of the enterprise's policies at each stage of development are given, which has strong practical significance.

## 6. Conclusion

The main work of this article is to research the integration and improvement path of enterprise green innovation capability. The essence of innovation integration in an enterprise is the effective integration and coordination of different knowledge subjects in the enterprise knowledge system. Different integration modes will form different innovation modes and achieve different innovation efficiencies. Therefore, this article will first determine the factors that affect the green innovation ability based on the knowledge niche integration mechanism and form a conceptual model by reviewing the hypothetical relationship between the factors in the literature construction. And through the model development strategy in the structural equation model, a sample model with practical significance is obtained to analyze the impact mechanism and intensity of different integration paths on green innovation capabilities. The final generation model of enterprise green innovation capability is obtained, and the mode of enterprise innovation integration is explored. This article studies the problem with the principles of scientificity, systematicness, and rigor, but there are still some deficiencies. Due to geographical restrictions, the heterogeneity in the sample is insufficient, and its research results may be different from enterprises in other regions.

The article "Integration of Green Innovation Capabilities of Enterprises Based on Ant Colony Optimization Algorithm" was retracted in 2023. Reasons: unreliable results or conclusions; concerns about the data; concerns about the peer review; concerns about the citations.

## Figures and Tables

**Figure 1:** The “knowledge niche” of two different types of firms.

**Figure 2:** Knowledge niche after corporate innovation integration.

**Figure 3:** Schematic diagram of the innovation system structure.

**Figure 4:** Business situation with different technology module types.

**Figure 5:** Integration of green innovation capabilities of enterprises in the same link.

**Figure 6:** Ant pathfinding.

**Figure 7:** Industry situation.

**Figure 8:** Regional distribution.

**Figure 9:** Reliability analysis results of green innovation influencing factors scale.

**Figure 10:** Table reliability analysis results of green dynamic capacity and green innovation capacity.

**Table 1:** Sample descriptive statistics.

		Number of companies	Mean	Standard deviation
Incremental innovation	Common technology modules	45	14.3	1.46
	Proprietary technology module	21	12.52	1.28

Breakthrough innovation	Common technology modules	45	9.25	2.0
	Proprietary technology module	21	12.74	1.68

**Table 2:** Independent samples test.

		*F* test	Salience	*t*-test	Salience	Average difference
Incremental innovation	Assuming equal variances	0.001	0.976	2.450	0.025	1.22
	Do not assume equal variances	—	—	2.368	0.019	1.22

Breakthrough innovation	Assuming equal variances	6.452	0.015	−3.848	0.000	1.79
	Do not assume equal variances	—	—	−3.780	0.000	1.79

**Table 3:** Measured model quality parameters in the revised model.

name	Item	Load	Significant level
Knowledge fusion ability	Q9	0.710	<0.001
	Q10	0.502	<0.001
	Q11	0.516	<0.001

**Table 4:** Measured model quality parameters in the revised model.

name	Item	Load	Significant level
Incremental innovation	Q53	0.884	<0.001
	Q54	0.630	<0.001
	Q55	0.918	<0.001
	Q56	0.654	<0.001

**Table 5:** Measured model quality parameters in the revised model.

name	Item	Load	Significant level
Breakthrough innovation	Q57	0.790	<0.001
	Q58	0.678	<0.001
	Q59	0.815	<0.001
	Q60	0.848	<0.001

## Data Availability

No data were used to support this study.
